The article "The Role of ET-1 in Early Cerebral Microcirculation Changes after Subarachnoid Hemorrhage" was retracted in 2023. Reasons: signs of a paper mill; suspected computer-generated content; unreliable results or conclusions; concerns about the data.

# The Role of ET-1 in Early Cerebral Microcirculation Changes after Subarachnoid Hemorrhage

**DOI:** 10.1155/2022/4592986

**Published:** 2022-04-11

**Authors:** Lei Qin, Yanan Wang, Zongyu Xie, Yichuan Ma

**Affiliations:** ^1^Department of Radiology, The First Affiliated Hospital of Bengbu Medical College, Bengbu 233000, China; ^2^Department of Medical Imaging Diagnostics, College of Medical Imaging, Bengbu Medical College, Bengbu 233000, China; ^3^Department of Function, The Second Affiliated Hospital of Bengbu Medical College, Bengbu 233040, China

## Abstract

Subarachnoid hemorrhage (SAH), especially aneurysmal subarachnoid hemorrhage, is a serious cerebrovascular disease with high mortality and morbidity. However, there is no effective treatment in clinics. In recent years, more and more studies have shown that early brain injury (EBI) may be an important reason for poor prognosis of SAH. Explore the mechanism of early brain injury after subarachnoid hemorrhage (SAH). In this study, 20 male New Zealand white rabbits were selected and divided into the experimental group and sham operation group, with 10 rabbits in each group. The neurobehavioral scores, food intake, and cerebral perfusion parameters, cerebral blood volume (CBV), cerebral blood flow velocity (CBF), ET-1, IL-1, and IL-6, in rabbit plasma were compared. The food intake scores and neurological dysfunction scores of the experimental group at 1 h, 6 h, 24 h, and 72 h after modeling were higher than those of the sham operation group, which had a statistical significance (*P* < 0.05). The dysfunction scores all showed a gradual decrease; the CBV and CBF values of the experimental group at 1 h, 6 h, 24 h, and 72 h after modeling were all lower than those of the sham operation group, which had a statistical significance (*P* < 0.05), and the MTT values were all higher than that of the sham operation group, which had a statistical significance (*P* < 0.05). The TTP values of rats in the experimental group were higher than those in the sham operation group at 6 h, 24 h, and 72 h after modeling (*P* < 0.05), the experimental group was in the modeling. The levels of serum ET-1, IL-1, and IL-6 at 1 h, 6 h, 24 h, and 72 h were higher than those in the sham operation group, which had a statistical significance (*P* < 0.05). New Zealand white rabbits can have brain perfusion volume disorder, inflammatory reaction, and cerebral vasospasm in the early stage after SAH, and brain injury can appear in the early stage.

## 1. Introduction

Subarachnoid hemorrhage (SAH) is a common clinical neurological disease caused by the rupture of blood vessels at the bottom of the brain or on the surface of the brain and spinal cord. The common causes include trauma and aneurysm, and the mortality and disability rate are extremely high [1, 2]. Early brain injury (EBI) caused by SAH involves a variety of pathophysiological changes such as vasospasm and delayed cerebral ischemia. The mechanism is complex and is related to the prognosis of patients. As blood enters the subarachnoid space, the intracranial pressure increases and the cerebral perfusion pressure decreases. The ischemic and anoxic state of the brain tissue can indirectly damage the vascular wall, thus forming microthrombosis, leading to brain cell edema and death [3]. In addition to the mechanical damage of blood to brain tissue, nitric oxide (NO) affects the resistance of brain microcirculation by dilating blood vessels, endothelin-1 (ET-1), inflammatory factors interleukin-1 (IL-1) and interleukin-6 (IL-6) affecting the blood vessel wall and blood-brain barrier (BBB), resulting in edema and necrosis of brain cells [4, 5]. Traditional examination cannot accurately reflect the state of cerebral microcirculation; noninvasive CT perfusion imaging can be through blood volume (CBV), blood flow (CBF), mean transit time (MTT), time to peak (TTP), and other parameters, showing the whole brain microcirculation in different lobes, especially ischemic brain tissue. In this study, CT whole brain perfusion imaging technology was used to simultaneously measure the changes of influencing factors such as ET-1, and the pathological changes of brain tissue were compared to observe the changes of brain microcirculation [6, 7]. Further understanding of the mechanism of SAH, with a view to clinical treatment of microcirculation changes as the basis for SAH treatment, reduces the mortality and disability rate.

The article "The Role of ET-1 in Early Cerebral Microcirculation Changes after Subarachnoid Hemorrhage" was retracted in 2023. Reasons: signs of a paper mill; suspected computer-generated content; unreliable results or conclusions; concerns about the data.

The rest of this study is organized as follows: Section 2 discusses related work.  Section 3 shows the experimental results. The results are discussed in Section 4, and Section 5 concludes the study with summary and future research directions.

## 2. Materials and Methods

### 2.1. Experimental Animal

Twenty male New Zealand white rabbits were selected and divided into the experimental group and the sham operation group with 10 rabbits in each group. The indexes at 1 h, 6 h, 24 h, and 72 h in the two groups were detected, respectively. The weight range was 2.6–3.3 kg, and the average weight was 2.90 ± 0.20 kg. Rabbits aged 3–5 months. Feed at room temperature 22–25°C, light 12 h, standard pellet feed, drinking water for tap water, and each rabbit a cage.

### 2.2. Establishment of the SAH Animal Model

Autologous arterial blood was injected into the cistern magna twice [8]. Specific operation: rabbits were placed in prone position and anesthetized with combined medication (0.1 mL/kg Sumianxin and 1 mL/kg pentobarbital sodium), iodophor disinfection, and 2 cm long median incision on occipital trochanter. Separate the cervical tissue layer by layer bluntly, expose the skull, and inject the needle into the gap between the lower occipital segment and the atlas. Blood (1 mL/kg) was drawn from the central artery of the rabbit ear and injected into the cisterna magna. After injection, attention should be paid to preventing cerebrospinal fluid leakage, pressing with gauze in time, and suturing muscles and skin after spraying penicillin powder on the wound. After the above operation, the rabbit head was downward for about 30 min, so that blood around the basilar artery was evenly distributed. Repeat the procedure after 48 h.

The article "The Role of ET-1 in Early Cerebral Microcirculation Changes after Subarachnoid Hemorrhage" was retracted in 2023. Reasons: signs of a paper mill; suspected computer-generated content; unreliable results or conclusions; concerns about the data.

The standard of successful modeling: when blood is injected into the cisterna magna, when the operator feels less resistance, that is, “sense of emptiness,” the puncture needle breaks through the dura, and when blood is injected into the cisterna magna, the rabbit breathes significantly deep and fast. CT scan showed high-density hemorrhage around the cistern magnum.

Neurological score of the SAH rabbit model before CT perfusion scanning, the reference standard, is as follows: whether standing, walking, and righting reflex reaction, score criteria were as follows: 0, normal; 1, mild damage; 2, moderate damage; 3, severe damage. Abdominal and dorsal reaction assessment scores were as follows: 0, normal; 1, restlessness; 2, open; 3, convulsion. The total blind scoring method was used to record the scores, and the total scores of each nervous system were taken to finally evaluate the overall neurological status.

### 2.3. Brain Perfusion Parameter Scanning

The GE revolution CT of the Radiology Department of the First Affiliated Hospital of Bengbu Medical College was used to collect perfusion imaging and hemodynamic parameters. After anesthesia, the contrast agent was injected through ear vein (iodophenol, 1.5–2.0 mL/kg). Scanning while administration, a total of 4000 images were collected, scanning interval 2 s, 120 kVp and 100 mA, image matrix 512 × 512, layer thickness 0.5 mm, and FOV 180 mm. Perfusion scan time was 55 s.

### 2.4. Methods for Specimen Collection and Detection

After CT perfusion scanning was completed, the animals were deeply anesthetized, and 500 mL 10% formalin was injected into the left ventricle. After about 30 min, the brain was removed by craniotomy. The brain tissue was taken symmetrically from each lobe of the brain, about 1 cm*∗*1 cm in size, fixed with paraformaldehyde for 2 days, paraffin embedded, and sliced after dehydration. Observe the changes of brain cells.

The article "The Role of ET-1 in Early Cerebral Microcirculation Changes after Subarachnoid Hemorrhage" was retracted in 2023. Reasons: signs of a paper mill; suspected computer-generated content; unreliable results or conclusions; concerns about the data.

Determination of ET-1 plasma content: enzyme-linked immunosorbent assay (ELISA) was used to add samples according to the instructions of the rabbit endothelin-1 (ET-1) ELISA kit. The absorbance of the microplate reader was read at 450 nm, and the sample concentration was calculated.

### 2.5. Observation on Food Intake and Neurological Dysfunction Score

All rabbits were fed with standard pellet feed and tap water, and the changes of food intake after modeling were observed and recorded. Endo four classification method scores are as follows: 1 point, no change in food intake and before modeling; 2 points, the food intake of rabbits reached >50–90% compared with that before modeling; 3 points, the food intake of rabbits was less than 50% before modeling; 4 points, no food at all.

After modeling, the neurological function of rabbits was recorded and scored according to the endo neurological function score method [9]. According to the movement and neurological status of rabbits on the flat ground, the scores were as follows: 1 point, there was no change in activity compared with before modeling; 2 points, there were mild or suspicious neurological dysfunction in rabbits (mainly manifested as poor spirit, drowsiness, malaise, rigidity of neck, reduced movement, slow reaction, and disordered hair); 3 points, moderate neurological dysfunction (such as chewing disorder and limb paralysis) occurred in rabbits; 4 points, rabbits showed severe neurological dysfunction (circle movement, walking difficulties, and limb paralysis).

### 2.6. Statistical Processing

In this study, the measurement indexes such as food intake, neurological deficit score, and cerebral perfusion parameters of rabbits were tested by normal distribution, which were in accordance with the approximate normal distribution or normal distribution, and expressed as ($\bar{x}$ ± *s*). The repeated measurement variance analysis was used for comparison between groups, and the LSD-*t* test was used for pairwise comparison between groups. Professional SPSS 21.0 software was used for data processing, test level *α* = 0.05.

## 3. Results

### 3.1. Comparison of Feeding Volume and Neurological Dysfunction Scores between the Two Groups

The food intake score and neurological dysfunction score of the experimental group were higher than those of the sham operation group at 1 h, 6 h, 24 h, and 72 h after modeling and which had a statistical significance (*P* < 0.05). The food intake score and neurological dysfunction score of the experimental group were gradually decreased, as shown in Figure 1.  Table 1 provides food intake and neurological dysfunction scores of the two groups.  Figure 2 shows trend chart of food intake score changes.  Figure 3 shows trend chart of neurological dysfunction score.

The article "The Role of ET-1 in Early Cerebral Microcirculation Changes after Subarachnoid Hemorrhage" was retracted in 2023. Reasons: signs of a paper mill; suspected computer-generated content; unreliable results or conclusions; concerns about the data.

### 3.2. Comparison of Cerebral Perfusion Parameters between the Two Groups of Animals

At 1 h, 6 h, 24 h, and 72 h after modeling, the CBV and CBF values in the experimental group were lower than those in the sham operation group, and the difference was statistically significant (*P* < 0.05). The MTT values were higher than those in the sham operation group, which had a statistical significance (*P* < 0.05).The TTP values at 6 h, 24 h, and 72 h after modeling in the experimental group were higher than those in the sham operation group (*P* < 0.05).  Table 2 provides comparison of changes in cerebral perfusion parameters of the two groups of animals.  Figure 4 shows CBV change trend chart.  Figure 5 shows CBF change trend chart.  Figure 6 shows MTT change trend chart.  Figure 7 shows TTP change trend chart.  Figure 8 shows the comparation of cerebral perfusion parameters between the two groups of animals.

### 3.3. Comparison of Serum ET-1, IL-1, and IL-6 Levels between the Two Groups of Animals

The levels of serum ET-1, IL-1, and IL-6 in the experimental group were higher than those in the sham operation group at 1 h, 6 h, 24 h, and 72 h after modeling, which had a statistical significance (*P* < 0.05).  Table 3 provides comparison of serum ET-1, IL-1, and IL-6 levels in the two groups of animals.  Figure 9 shows ET-1 change trend chart.  Figure 10 shows IL-1 change trend chart.  Figure 11 shows IL-6 change trend chart.

## 4. Experimental Data Analysis

SSAH is a serious cerebrovascular disease, and there is still a high mortality rate after drug and surgical treatment. Cerebral vasospasm and delayed cerebral ischemia are the main complications [10]. The concept of whole brain perfusion imaging proposed by Miles in 1991 has been widely used in neuromedicine [11]. This technique can distinguish and quantify the normal perfusion area, ischemic area, and infarct area of brain tissue in patients with brain injury and evaluate BBB permeability, which is one of the effective methods for the diagnosis of neurological diseases such as subarachnoid hemorrhage.

In this study, the time characteristics of CT perfusion parameters, food intake score, and neurological dysfunction score at 1 h, 6 h, 24 h, and 72 h after SAH were analyzed. The results showed that the experimental group was higher than that of the sham operation group. The food intake score and neurological dysfunction score of the experimental group showed a decreasing trend. The possible reason was acute vasospasm caused by surgical modeling, which did not cause long-term serious neurological symptoms and excluded delayed vasospasm but also did not exclude the existence of cerebral circulation compensation [12]. At 1 h, 6 h, 24 h, and 72 h after SAH, the CBV and CBF values of the experimental group were lower than those of the sham operation group, and the MTT value was higher than that of the sham operation group, indicating that the rabbit SAH model caused reversible and irreversible ischemic injury, which was consistent with the experimental requirements. MTT is the average time when the contrast agent passes through the capillary, which can be used as an effective indicator for judging brain ischemia [13]. 1 h, 6 h, 24 h, and 72 h after modeling, serum ET-1, IL-1, and IL-6 levels were higher than the sham group. This value is related to the occurrence of delayed cerebral ischemia. IL-1Ra, an IL-1 receptor antagonist, can block the upregulation of IL-6, which has been proved to prevent experimental-induced cerebral ischemia and traumatic brain injury [14]. At 6 h, 24 h, and 72 h after SAH, the TTP value of the experimental group was higher than that of the sham operation group. It also showed that the early brain injury such as cerebral perfusion disorder, inflammatory response, and cerebral vasospasm occurred in rabbits after SAH, which was consistent with expectations. ET-1 acts as an important regulator by binding to receptor ETA and ETB. ET-1 specifically binds to ETA, resulting in vasoconstriction and reduced blood flow. It can be seen in our experiment that SAH injury of endothelial cells leads to the release of ET-1 in large quantities, and the level of ET-1 in plasma also increases, and its content is positively correlated with SAH symptoms [15]. ET-1 does not change the resting CBF. When the blood-brain barrier is damaged, the increase of ET-1 level affects the cerebral vascular function. Injection of ETAR antagonist into the cistern can improve the blood perfusion after SAH [16, 17]. At present, the mechanism of ETR antagonist in the treatment of SAH is not clear, and more studies can be carried out in the future to improve the early brain injury after SAH [18].

The article "The Role of ET-1 in Early Cerebral Microcirculation Changes after Subarachnoid Hemorrhage" was retracted in 2023. Reasons: signs of a paper mill; suspected computer-generated content; unreliable results or conclusions; concerns about the data.

The results of this study showed that the concentration changes of ET-1, IL-1, and IL-6 in serum were effective indicators for SAH observation [19, 20]. In this study, New Zealand rabbits were used to establish models. Compared with rat or mouse models, the multiperiod serum extraction method was adopted. The extraction method was simple, and the success rate was high. The sample size was large, and the mortality and disability rate were low [21, 22]. It provided ideas for the study of serum-related protein expression after SAH and the detection and judgment of SAH severity by serum-related protein. In this experiment, according to the CT whole brain perfusion imaging map and the pathological changes of brain tissue slices, the temporal changes of brain microcirculation were analyzed to avoid the single use of CT whole brain perfusion imaging technology affected by single use of CT whole brain perfusion imaging technology, as well as the differences in CBF, CBV, MTT, and TTP values due to different equipment and technical operations, and the difficulty in reaching a consensus on the quantitative threshold of different equipment. Comprehensive indexes were used to analyze the brain injury and cerebral microcirculation after SAH, so as to reduce the error of single numerical judgment and become the basis for SAH treatment.

## 5. Conclusion

After SAH in the rabbit model, ischemic injury and inflammation led to decreased cerebral perfusion and microcirculation disturbance, affecting neurological dysfunction and limb coordination. CT perfusion parameters can be used to analyze the degree of ischemic injury. MTT can be used as one of the effective indicators to judge cerebral ischemia, combined with other indicators to reduce the judgment error. However, there is still a lack of cell experiments and clinical experiments to prove whether the related tissue cells cause the concentration changes of ET-1, IL-1, and IL-6 after SAH, whether the effect of antagonism or inhibition of the related tissue cells can inhibit the development of SAH by affecting CBF, CBV, MTT, and TTP, and whether the related antagonists or inhibitors can be put into clinical use to improve the prognosis of patients. In the future, we should further increase and improve the data of cell experiments and clinical experiments and comprehensively analyze the temporal changes and internal related mechanisms of CT whole brain perfusion imaging and ET-1 after SAH, so as to provide reference for clinical judgment of human SAH and subsequent treatment.

## Figures and Tables

**Figure 1:** (a) Animal model making. (b) Brain tissue extraction.

**Figure 2:** Trend chart of food intake score changes.

**Figure 3:** Trend chart of neurological dysfunction score.

**Figure 4:** CBV change trend chart.

**Figure 5:** CBF change trend chart.

**Figure 6:** MTTchange trend chart.

**Figure 7:** TTP change trend chart.

**Figure 8:** (a) Pseudocolor image of CT perfusion 72 hours after modeling in the model group (CBV is 4.70 mL/100 g, CBF is 274.81 ml/min/100 g, MTT is 1.74 s, and TTP is 9.28 s). (b) Brain tissue after modeling. Regular H&E staining (20 *μ*m) at 72 hours showed that a large number of inflammatory cells infiltrated around the bleeding lesion, and the nerve cell edema was obvious.

The article "The Role of ET-1 in Early Cerebral Microcirculation Changes after Subarachnoid Hemorrhage" was retracted in 2023. Reasons: signs of a paper mill; suspected computer-generated content; unreliable results or conclusions; concerns about the data.

**Figure 9:** ET-1 change trend chart.

**Figure 10:** IL-1 change trend chart.

**Figure 11:** IL-6 change trend chart.

**Table 1:** Food intake and neurological dysfunction scores of the two groups ($\bar{x}$ ± *s*, scores).

Index	Group	1 h	6 h	24 h	72 h
Food intake score	Test group (*n* = 10)	3.31 ± 0.67	3.10 ± 0.74	2.88 ± 0.58	2.40 ± 0.60
	Mock surgical group (*n* = 10)	1.49 ± 0.22	1.51 ± 0.24	1.43 ± 0.21	1.36 ± 0.25
	*t*	8.161	6.463	7.433	5.060
	*P*	0.001	001	0.001	0.001

Neurological dysfunction score	Test group (*n* = 10)	3.10 ± 0.69	3.02 ± 0.77	2.80 ± 0.75	2.54 ± 0.68
	Mock surgical group (*n* = 10)	1.20 ± 0.19	1.14 ± 0.20	1.25 ± 0.21	1.30 ± 0.28
	*t*	8.395	7.473	6.293	5.332
	*P*	0.001	0.001	0.001	0.001

**Table 2:** Comparison of changes in cerebral perfusion parameters of the two groups of animals ($\bar{x}$ ± *s*).

Index	Group	1 h	6 h	24 h	72 h
CBV (ml/100 g)	Test group (*n* = 10)	4.79 ± 0.98	5.17 ± 0.68	4.58 ± 0.77	4.76 ± 0.90
	Mock surgical group (*n* = 10)	8.02 ± 1.20	9.93 ± 2.48	10.95 ± 1.06	7.39 ± 2.98
	*t*	−6.593	−5.853	−15.375	−2.672
	*P*	0.001	0.001	0.001	0.016

CBF (ml/min/100 g)	Test group (*n* = 10)	353.71 ± 42.94	257.32 ± 37.25	182.15 ± 16.36	269.05 ± 41.86
	Mock surgical group (*n* = 10)	632.45 ± 95.69	657.52 ± 61.15	559.14 ± 104.30	550.79 ± 115.29
	*t*	−8.404	−17.675	−11.292	−7.264
	*P*	0.001	0.001	0.001	0.001

MTT (s)	Test group (*n* = 10)	1.76 ± 0.21	2.19 ± 0.43	2.70 ± 0.67	1.64 ± 0.64
	Mock surgical group (*n* = 10)	0.74 ± 0.29	0.87 ± 0.33	1.00 ± 0.42	1.00 ± 0.25
	*t*	9.009	7.701	6.798	2.946
	*P*	0.001	0.001	0.001	0.009

TTP (s)	Test group (*n* = 10)	9.02 ± 0.78	9.25 ± 1.13	9.01 ± 0.99	9.07 ± 0.46
	Mock surgical group (*n* = 10)	8.25 ± 1.09	7.85 ± 0.83	7.73 ± 0.58	8.31 ± 0.71
	*t*	1.817	3.158	3.528	2.841
	*P*	0.086	0.005	0.002	0.011

**Table 3:** Comparison of serum ET-1, IL-1, and IL-6 levels in the two groups of animals ($\bar{x}$ ± *s*).

Index	Group	1 h	6 h	24 h	72 h
ET-1 (ng/mL)	Test group (*n* = 10)	35.96 ± 5.80	51.53 ± 7.91	70.59 ± 3.42	93.97 ± 11.61
	Mock surgical group (*n* = 10)	24.78 ± 5.12	23.44 ± 3.39	25.30 ± 4.59	44.04 ± 9.29
	*t*	4.570	10.322	25.021	5.674
	*P*	0.001	0.001	0.001	0.001

IL-1 (pg/mL)	Test group (*n* = 10)	61.14 ± 9.73	86.88 ± 3.51	117.43 ± 10.34	185.61 ± 55.05
	Mock surgical group (*n* = 10)	27.57 ± 5.65	30.92 ± 2.26	32.99 ± 5.35	30.69 ± 3.54
	*t*	9.435	42.389	22.936	8.881
	*P*	0.001	0.001	0.001	0.001

IL-6 (pg/mL)	Test group (*n* = 10)	67.86 ± 11.33	73.81 ± 13.87	111.73 ± 10.02	198.06 ± 15.32
	Mock surgical group (*n* = 10)	38.05 ± 8.94	32.18 ± 5.11	33.79 ± 3.62	30.97 ± 2.15
	*t*	6.532	8.906	23.134	34.155
	*P*	0.001	0.001	0.001	0.001

The article "The Role of ET-1 in Early Cerebral Microcirculation Changes after Subarachnoid Hemorrhage" was retracted in 2023. Reasons: signs of a paper mill; suspected computer-generated content; unreliable results or conclusions; concerns about the data.

## Data Availability

The data used to support the findings of this study are available from the corresponding author upon request.
